RETRACTED

# Application of the Improved Clustering Algorithm in Operating Room Nursing Recommendation under the Background of Medical Big Data

**DOI:** 10.1155/2022/4299280

**Published:** 2022-03-23

**Authors:** Xiaofang Wu, Chunjun Wang, Fangzhen Cai, Yingfen Wu

**Affiliations:** ^1^The Second Affiliated Hospital of Hainan Medical College, Haikou 570311, China; ^2^Hainan Women and Children's Medical Center, Haikou 570000, China

## Abstract

The nursing work in the operating room has the characteristics of long time, strong technicality, and heavy work, which have an important influence on the quality of the operation. Operating room nursing recommendations based on data mining technology can solve a series of practical problems in clinical nursing and nursing management. This paper selects the clustering algorithm in commonly used data mining technology as the research object and actually analyzes the impact of this algorithm in operating room nursing recommendations. At this stage, there is little research on data mining technology in the field of nursing in China. This paper aims to provide new ideas for the field of nursing research by exploring the actual application in the field of nursing.

## 1. Introduction

In the traditional medical process, medical resources such as medical staff are randomly allocated, which not only causes a waste of limited medical resources but also may delay the optimal treatment time for patients. With the development of science and technology, data mining technology as an emerging data analysis method has been widely used in various industries. The rapid development of medical informatization has led to the exponential growth of medical data, and the growth of medical big data has also placed a huge burden on the existing information systems of hospitals. For all kinds of unstructured medical data, the hospital information system cannot meet the requirements in terms of information processing speed, resulting in a lot of waste of valuable medical data.

The well-known consulting company pointed out in the report [1] released in 2011 that “Big data is the guideline to promote future productivity development, innovation, and consumer demand.” The International Data Center defines big data and attributes it to data with characteristics such as high capacity, diversity, high speed, and low value density [2]. The National Institute of Standards and Technology of the United States believes that big data refers to data capacity, data acquisition speed, or data representation that restricts the analysis and processing capabilities of traditional relational methods and requires the use of expansion mechanisms to improve processing efficiency. It is not difficult to see that different expert organizations have different definitions of big data, but they all define it from the perspective of data characteristics and emphasize the data processing methods.

RETRACTED

Medical big data retains the basic characteristics of big data. The biggest feature is diversity and redundancy. Therefore, at this stage, the hospital information system cannot process medical information data efficiently, and it significantly increases medical costs. Medical big data mainly comes from health data generated by healthcare systems, biomedicine, molecular medicine, social media, and sensors. Medical big data [3] has a wide range of sources, complex coverage, diverse structures, and fast update speeds, which also indirectly increase medical costs.

Nursing big data mainly includes clinical research data, various management data, various registration records (medical insurance registration, birth and death registration, and chronic and infectious disease registration), and admission registration and electronic health records, which contain a large amount of nursing data. Some experts also believe that nursing big data generally refers to data related to nursing and life and health, including patient vital signs, disease changes, and various test indicators. However, nursing big data emphasizes the nursing methods used by nurses to care for patients and improve their health. The medical information system needs to process nursing big data efficiently to improve nursing methods and improve the quality of care.

With the advent of the era of informatization “smart medical care” [4] and the use of efficient, convenient, and intelligent big data analysis and processing software to accurately identify patients and optimally allocate nursing doctors to improve the quality of care in the operating room, clustering algorithms have received significant attention.

## 2. Clustering Algorithm

The clustering algorithm [4] divides the dataset into several parts according to the idea of “things are clustered together,” and the data in each part has a high degree of similarity. Cluster analysis is an important algorithm component of current data mining technology. So far, related scholars have proposed a variety of improvements based on clustering algorithms. In the field of machine learning, clustering algorithms belong to unsupervised learning. Unlike classification, unsupervised learning does not rely on preset categories and training examples with class labels. Therefore, clustering belongs to observational learning rather than instance learning.

Many clustering algorithms cluster digital data, but in practical applications, other types of data (ordinal and binary data) need to be clustered. Common cluster analysis applications require users to input certain parameters to determine the number of clusters. Because the clustering results are very sensitive to the input parameters, it is difficult to determine, especially for datasets containing high-dimensional objects. Therefore, it is very important to study algorithms that are not sensitive to the order of data input. Essentially, the clustering algorithm is an optimization iterative process; through iterative operations, the objective function can get an optimal solution. But often the objective function is a nonconvex function in space [5]; with many minimums, only one is a global minimum, and the others are local minimums. The goal of optimization is to achieve global optimization and improve the existing clustering algorithm to be able to perform incremental clustering and have good scalability.

RETRACTED

### 2.1. Algorithm Based on Distance

The goal of cluster analysis is to classify similar instances into discontinuous groups, and the distance between two instances needs to be approximated. In cluster analysis, mathematical distance measurement is used to determine the degree of dissimilarity between two individuals. There are many distance-based measurement methods available, and the most familiar is the Pearson correlation coefficient method. Euclid's straight-line distance is based on Pythagoras's theorem. Manhattan distance [6] is the sum of the projection distances of the line segment formed by two points on the fixed rectangular coordinate system of the Euclidean space to the axis. It is a commonly used distance-based clustering analysis algorithm in data mining technology. K-means is a typical distance-based clustering algorithm that uses distance as the evaluation criterion of similarity. The greater the distance between two objects, the higher the similarity. K-means clustering requires the user to specify a cluster number *k* as the prerequisite input data. The selection of K initial clustering center points has a greater impact on the clustering results, so it is generally necessary to estimate the value of *k* in advance to achieve high-quality clustering.

The algorithm steps are as follows:

1. Immediately select any *k* objects as the initial cluster center, which initially represents a cluster
2. Calculate the distance from the point to the centroid and classify it into the class of the nearest centroid
3. Recalculate the centroid of each class
4. Iterate 2∼3 steps until the centroid is equal to the original centroid or less than the specified threshold

### 2.2. Density-Based Algorithm

Density-based clustering analysis classifies data objects according to whether they belong to connected density domains. The commonly used density-based clustering algorithm is DBSCAN [7]. It is generally assumed that the category can be determined by the tightness of the sample distribution. The samples of the same category are closely connected, and there must be samples of the same category not far from any sample of the category.

RETRACTED

The algorithm steps are as follows:

  Input: sample set *D*={*x*_1_, *x*_2_,…, *x*_*m*_}; neighborhood parameter (*ε*, MinPts).
(1) Initialize the core object set Ω, ≠0; initialize the category *k* = 0.
(2) Traverse the elements of *D*; if it is a core element, add it to the core object set Ω.
(3) If all the elements in the core object set Ω have been accessed, the algorithm ends; otherwise, go to step 4.
(4) In the core object Ω, immediately select an unvisited core object *o*, first mark *o* as visited, then mark *o* as category *k*, and finally store the unvisited data in *o*'s *ε* in the seed set Seeds.
(5) If the seed set *See*  *ds*  !=0, the current cluster has been generated and  *k*=*k*+1 jumps to 3. Otherwise, select a seed point from the seed set Seeds, first mark it as visited, mark category *k*, and then judge whether the seed is a core object; if it is to add unvisited seed points in the seed to the seed set, jump to 5.

### 2.3. Model-Based Algorithm

The model-based clustering algorithm is to find the data to best fit the preset model for each class. The commonly used model-based clustering algorithm is the COBWEB [8] algorithm. Clustering is mainly for noun-type data. The input objects are described by classification attribute-value pairs, and hierarchical clustering is created in the form of a classification tree. The histogram formed in the COBWEB algorithm is called a classification tree, and each node in the classification tree corresponds to a concept. This concept describes information such as the probability of the object being classified under the node and the conditional probability of the attribute-value pair. In the construction of the classification tree, each new object moves down the tree species along the path of the “best” matching node and is classified, and the classification tree is constantly updated. This process is guided by classification utility. The COBWEB algorithm is faster, but it needs to assume that the probability distribution on each attribute is independent of each other, and it may lead to a highly imbalanced classification tree.

## 3. Application of Machine Learning Algorithms

In operating room nursing recommendations, clustering algorithms can help nurses and other medical staff distinguish patients from the hospital information management system, discover deeper information about each type of patient by using data mining and analysis methods, summarize the individual characteristics and clinical features of each type of patient, check the characteristics, and provide targeted treatments for patients, thereby reducing the psychological and financial burden of patients and improving the quality of life of patients.

RETRACTED

### 3.1. Algorithm Analysis and Comparison

Decision tree has carried out relevant research in clinical nursing and nursing management. Park et al. used a decision tree combined with logistic regression and support vector machine [9] to analyze the electronic health record data of a hospital to determine the risk factors of catheter-related urinary tract infection. Duriakova et al. [10] used decision tree combined with artificial neural network and support vector machine algorithm to establish a prediction model of urinary tract infection. This model has an accuracy rate of 98.3% for the diagnosis of urinary tract infection, which provides clinically targeted nursing work. Lisi et al. [11] used decision trees to analyze the bed-to-care ratio and nursing work indicators in 22 wards and deployed nurses in the ward based on the results. The results of the deployment were achieved in terms of objectivity, applicability, and acceptance. The results show the satisfaction and approval of 45 nursing managers. Zuo Fenghua applied the decision tree analysis method to nursing quality management. Based on the data of 390 nurses and the survey results of 585 patients on nursing work quality evaluation, a model is established, and an evaluation system is constructed after comprehensive analysis so as to evaluate each ward in a fair and just manner.

Decision tree is mainly used in the clinical nursing research that has been carried out to analyze the related influencing factors of a clinical symptom and the establishment of related models to find the main risk factors and strengthen the nursing care in a targeted manner [12]. It has been applied to nurse resource allocation and nursing quality assessment in nursing management work [13]. The implementation of the decision tree is helpful for nursing staff not only to analyze the influencing factors of various clinical symptoms but also to implement targeted nursing measures based on the analysis results, thereby effectively reducing patient complications and improving the quality of care [14]. It can also be used to establish predictive evaluation models to support clinical decision-making, thereby reducing medical costs and saving medical resources [15]. However, comparing domestic and foreign studies, it is found that foreign countries often combine decision trees with other data analysis methods to solve patient-related problems, while domestic studies often apply single decision tree methods to issues such as nursing resource allocation and nursing quality management. There are relatively few studies on patient-related issues.

RETRACTED

Clinical nursing and nursing teaching have been involved in nursing research. Chiang et al. investigated and clustered the symptoms of 75 patients with systemic lupus erythematosus and clarified the focus and direction that nursing staff should pay attention to. Chow et al. clustered analysis on the clinical skills, knowledge, attitude, and perception ability of 253 nursing students about hospice care, and the results showed that clinical experience is an important factor affecting the ability and attitude of nursing students in hospice care. Li Caifen and others analyzed 681 medical records of patients with hypertension by clustering and discovered the common nursing diagnosis of hypertension patients and the main reasons for poor blood pressure control, thereby instructing specialist nurses to improve the quality of care. Wu Ning et al. analyzed the key fields of PubMed's tumor care literature from 2008 to 2017 by two-way clustering and established a word frequency matrix to explore the development trend of tumor care research. Cluster analysis is widely used in nursing-related research, and clinical research focuses on the clinical symptoms of diseases to understand the symptom clusters of various diseases and provide targeted interventions in clinical nursing work. Empirical evidence is used in the teaching and education management of nursing students, which is conducive to the setting and arrangement of students' courses; when used in nursing research, it can provide direction for the development trend of nursing specialty research [16]. However, in our country, cluster analysis is mainly applied to the visualization analysis of the literature and the metrological analysis of various fields of nursing to reveal the current research trends and focus and to discover the weak areas of current research and grasp the latest developments in nursing research. And the overall characteristics provide a reference for further research.

The prerequisite of the model-based clustering algorithm requires that each attribute of the analysis object is independent and identically distributed, but this is an ideal state [17]. Density-based and distance-based clustering algorithms require users to set certain parameters in the early stage to produce acceptable clustering results [18]. Different initial values often lead to different clustering results, usually local optimal solutions. In fact, this type of algorithm generally requires an exhaustive list of all possible divisions in practical applications [19].

RETRACTED

Reasonable clustering of patient care data based on individual patient parameters is different from cluster analysis in other fields. First, the individual patient characteristic data does not satisfy an independent probability distribution, and the deviation of a certain index often depends on other characteristics; second, certain parameters are often set to produce acceptable clustering results in the early stage of nursing, which requires rich medical experience and a certain degree of computer theory knowledge. Third, the actual conditions of patients vary greatly, making it difficult to choose a suitable value, and the actual operability is low.

### 3.2. Application of the Improved Clustering Algorithm

In order to improve the nursing efficiency of the operating room in the hospital, strengthen the construction of the nursing team in the operating room, and provide the basis for training of specialist nurses in the operating room and the reference basis for optimizing the operation process, this paper uses an improved clustering algorithm to comprehensively evaluate the efficiency of nursing human resources in the operating room.

The research content is as follows:

1. Investigate the current situation of human resource allocation in the operating room of the hospital, and use the questionnaire to understand the size of the operating room, the ratio of nurses, the number of administrative assistants, the number of logistic personnel, the training status of specialist nurses, the social status of each respondent, demographic characteristics, and so on and give analysis
2. Investigate the time interval and interstage interval of the first operation in the nine operating rooms, measure and analyze the effective nursing hours, and provide a reference for improving the utilization rate of the operating room and the efficiency of nursing staff
3. Use clustering algorithm to evaluate the nursing efficiency of operating rooms in nine hospitals, find out the operating rooms with relatively low nursing efficiency, and calculate the ideal value of various nursing input indicators and output indicators under the current scale conditions

According to the current medical big data background, the hierarchical improved clustering algorithm [16] is more suitable for scientific and efficient operating room nursing recommendation applications because the hierarchical clustering algorithm requires fewer prerequisites and a hierarchical nested tree.

The algorithm steps are as follows:

  Suppose there are *n* samples to be clustered
(1) Initialization: treat each sample as a cluster
(2) Calculate the similarity between each cluster
(3) Find the nearest two clusters and classify them into one category
(4) Repeat Steps 2 and 3 until all samples are classified into one category

The whole process is to build a hierarchical nested tree. In the process of building, you can set the number of categories that need to be classified in Step 4.

RETRACTED

In the application process of operating room care recommendations, treat each patient as a category. Use Manhattan distance, Chebyshev distance, and other methods to calculate the similarity between each category; clustering ends when the similarity is greater than a certain termination condition.

The working hours' measurement method was used to determine the effective nursing working hours per day per capita in each operating room. First, investigate and understand the work content of each shift in the operating room, refer to the experience questionnaire, and then combine the specialty characteristics of the operating room with a head nurse who has worked in the operating room for more than 20 years to design the operating room nursing project time measurement questionnaire. After two rounds of discussion by four operating room nursing experts and two nursing management experts, the decision was made based on the preinvestigation information feedback questionnaire.  Figure 1 is the technology line.

Questionnaires are self-designed for head nurses and nurses in the operating room. Both questionnaires include some sociodemographic characteristics of the respondents (age, ethnicity, highest education, professional title, and working experience). The head nurse questionnaire also involves the number of nurses in 2011, proportion of nurses' professional titles, operating room, ratio of desk nurses, number of male nurses, number of administrative support staff, number of logistics staff, training of specialist nurses, per capita annual income of nurses, nursing consumables, number of emergency surgeries per year, number of surgeries per year, average per day information such as the number of sets, and nursing business income. The content of the nurse questionnaire involves information about whether or not they have been trained by specialist nurses in the operating room and the training time and the reason why the first operation could not start on time.

Index of content validity (CVI ) refers to the agreement between the content measured by the questionnaire and the content to be measured. The three self-made questionnaires in this study were formulated with reference to relevant literature. Before the investigation, they passed the examinations of 4 operating room nursing experts (1head nurse, 3 deputy head nurses, 2 university and undergraduate nurses) and 2 nurses. Management experts (all are chief nurses, one for college and one for undergraduate) use the item evaluation form of the 4-point relevance assessment, the three self-made questionnaires in this study are evaluated, and the CVI values are 0.960, 0.924, and 0.851.

RETRACTED

The content reliability of the questionnaire is assessed using Cronbach's alpha, which represents the consistency between the scores of each item in the questionnaire. This study used convenient sampling to select 24 (4 head nurses and 20 nurses) qualified operating room nurses to conduct preinvestigation on three self-made questionnaires and test the reliability of the results. The measured Cronbach coefficients were 0.895, 0.854, and 0.801, respectively. It is generally believed that the reliability is better when the coefficient is greater than 0.7.

By consulting a large number of relevant domestic and foreign pieces of literature, referring to the experience questionnaire, and combining the special features of the operating room, we designed the questionnaire with a head nurse who has worked in the operating room for more than 20 years. Timely adjust and improve the questions in the questionnaire through presurveys, and test the reliability and validity of the questionnaire. The “Operating Room Head Nurse Questionnaire,” “Operating Room Nurse Questionnaire,” and “Working Hours Questionnaire” were sent to 6 experts for review before the investigation. Among them, 4 were operating room nursing experts (1 head nurse, deputy director, and 3 nurses, 2 are junior college and undergraduate), and 2 are nursing management experts (both head nurses), and 1 is junior college and undergraduate. The measured CVI values are 0.960, 0.924, and 0.851, respectively. After a preliminary investigation, the Cronbach coefficients were 0.895, 0.854, and 0.801, respectively. It is suggested that this questionnaire has good reliability and validity.

A total of 9 questionnaires for head nurses in the operating room were issued in this survey, and 9 copies were recovered, with a recovery rate of 100%. There are 9 valid questionnaires, with an effective rate of 100%. A total of 310 questionnaires for nurses in the operating room were issued, and 292 valid questionnaires were returned, with an effective rate of 94.19%. There were 292 operating room nurses surveyed, with an average age of 28.92 ± 6.51 years. There are 15 head nurses with an average age of 41.13 ± 6.83 years and 2 chief nurses, 4 deputy chief nurses, 5 supervisor nurses, 4 nurses, 6 undergraduates, and 9 junior college nurses. According to the data provided by the head nurses of the operating rooms of the nine hospitals, there are a total of 413 operating room nurses (including the head nurses), of which 38 male nurses account for 9.20%, and those who do not have a master's degree.  Table 1 shows general information for operating room nurses.

RETRACTED

According to the data provided by the head nurses of the operating rooms of each hospital, there are a total of 583 total staff (nurses and logistics staff) in the operating rooms of the 9 hospitals, a total of 413 nurses, a total of 170 logistics staff, a total of 154 open operating rooms, and a total of 154 operating rooms. There are 38 administrative staff, and the specific statistics of each hospital are shown in Table 2.

Nursing workload is the basis for nursing cost accounting and the main basis for the deployment of nursing staff. Nursing hours are the sum of the time required to complete each nursing item, that is, the amount and proportion of direct and indirect nursing hours. Direct nursing hours refer to the nursing, treatment, education, and other service hours directly provided by nurses to patients, such as posture and preoperative visits. Indirect nursing hours refer to not directly serving patients or preparing for direct nursing, as well as communication and coordination. It takes time to prepare indirect nursing, such as placing sterile operating table, brushing teeth, coordinating department work, etc.

The standard deviation is used to indicate that the daily effective nursing working hours of all nurses in the operating rooms of 9 hospitals are 345 min, direct nursing working hours are 201 min, accounting for 58% of the daily effective nursing working hours per capita, and indirect nursing working hours are 1431 min. It accounts for 41% of the effective nursing hours per capita per day. Other conditions are shown in Table 3.

The basic situation of the actual data before and after the improvement of the optimization algorithm in the operating rooms of each hospital is shown in Table 4.

The use of the improved clustering algorithm is a novel nursing method of operating room nursing, which can systematically optimize the nursing process through scientific methods during the operation of the patient, further improve the efficiency of nursing work, and greatly reduce the errors in the nursing process, thereby ensuring the quality of the operation and improving the patient's satisfaction with the operation. Before the operation, the relevant nursing staff should communicate effectively with the patient and family members, fully grasp the patient's condition and other pieces of information, answer the patient's questions about the operation in a timely manner, and conduct comprehensive nursing interventions according to the actual situation of the patient to ensure that the patient is always in the best position during the operation. In addition, operating room care using an improved clustering algorithm can eliminate the inexplicable fear and tension of patients during the operation and eliminate the patient's interference by other factors. At the same time, after the patient's operation, the nursing staff can effectively prevent adverse reactions and complications for the patient according to the nursing recommendations and also assess the risk of postoperative complications and take preventive measures for the patient in time. In actual nursing management, broadly speaking, the scope of nursing management staff includes not only hospital nurses and family nurses but also experts and doctors. In traditional nursing management, experts, resident doctors, and nurses are randomly assigned and combined, which often produces different treatment effects and medical expenses. In order to improve this situation, some scholars have begun to discuss optimizing the nursing process and improving the nursing model to improve the quality of nursing. However, although these methods have improved the quality of care to some extent, they are less targeted. Therefore, in the analysis of nursing management, it can be considered in advance to simulate the treatment effect of different doctors on each patient. Use cluster analysis method to classify patients scientifically, comprehensive cluster results, patient's final cure status, and medical expenses, and find the best caregiver for each type of patient, so as to provide a certain reference basis for the hospital to carry out scientific nursing management. It can be seen that the operating room nursing recommendation based on the improved clustering algorithm is of great significance to surgical work.

RETRACTED

## 4. Conclusion

With the continuous advancement of public hospital reforms and the in-depth development of high-quality nursing services, the content and service mode of nursing work in the operating room is no longer based on cooperating with the doctor to complete the operation but requires the nurses in the operating room to go to the ward to perform preoperation for patients nursing services such as visits and postoperative return visits; therefore, the recommended configuration of operating room nursing has become a concern of current nursing managers. In summary, data mining technology based on the improved clustering algorithm can effectively improve the quality of care during the nursing period in the operating room, obviously can stabilize the various indicators of the patient during the operation, greatly improve the negative emotions of the patient, and increase the satisfaction of nursing work.

## Figures and Tables

**Figure 1:** Technology line.

**Table 1:** General information for operating room nurses.

Item	Group	General nurse		Nurse practitioner	
		Number (*n*)	Composition ratio (%)	Number (*n*)	Composition ratio (%)
Age	<30	212	72.60	0	0
	30∼40	62	21.20	9	60.00
	>41	18	6.20	6	40.00

Ethnicity	Han Chinese	213	72.90	14	93.33
	Ethnic minority	79	27.10	1	6.67

Academic qualifications	College	42	14.40	0	0
	Junior college	192	65.85	9	60.00
	Undergraduate	58	19.90	6	40.00
	Master	0	0	0	0

Title	Junior	239	81.80	4	26.67
	Intermediate title	50	17.10	5	33.33
	Senior title	3	1	6	40.00

Years of work	<3	89	30.50	0	0
	4∼10	130	44.50	0	0
	11∼20	51	17.50	8	53.33
	>21	22	7.50	7	46.67

Nurse training	True	229	78.40		100
	False	63	21.60		

**Table 2:** Open operating rooms, number of nurses, desk-to-nurse ratio, and administrative staff in each hospital operating room.

Hospital	Total	Nurses	Logistics	Operating rooms	Table-nursing ratio	Male nurses	Administrative support	
							Staff	Percentage
1	212	136	76	46	1/3	22	11	8.09
2	110	79	31	30	1/2.6	5	9	11.39
3	59	45	14	18	1/2.5	2	2	4.44
4	26	21	5	10	1/2.1	0	1	4.76
5	52	39	13	14	1/2.2	6	2	5.13
6	28	22	6	10	1/2.2	0	3	13.674
7	10	9	1	5	1/1.8	2	1	11.11
8	48	36	12	12	1/3.0	1	1	2.78
9	38	26	12	9	1/2.9	0	3	11.54

**Table 3:** Nursing hours per day per operating room nurse by hospital.

Hospital	Effective nursing hours per capita per day	Direct nursing hours	Composition ratio
1	288	170	59
2	347	180	51
3	402	229	57
4	280	162	57
5	426	240	56
6	181	102	56
7	191	105	55
8	325	206	63
9	322	210	65

**Table 4:** Actual data of comparison scores before and after improvement of the optimization algorithm in operating rooms of each hospital.

Operating room	Number of nurses		Effective nursing hours per day	
	Before optimization	After optimization	Before optimization	After optimization
1	65	79	267	322
2	35	45	256	325
3	19	21	211	402
4	14	22	129	191
5	6	9	73	280
6	75	85	243	323
7	36	55	167	256
8	33	45	126	189
9	23	41	104	156

## Data Availability

The simulation experiment data used to support the findings of this study are available from the corresponding author upon request.
